The article "Analysis of the Role of Comprehensive Treatment Model in the Treatment of Prostate Cancer" was retracted in 2023. Reason: concerns about the peer review.

# Analysis of the Role of Comprehensive Treatment Model in the Treatment of Prostate Cancer

**DOI:** 10.1155/2022/2118823

**Published:** 2022-01-05

**Authors:** Shuai Yang, Han Guan, Zhijun Chen, Sheng Wang, Hongliang Wu, Weide Zhong

**Affiliations:** ^1^Jinan University, Guangzhou, Guangdong 510632, China; ^2^Department of Urology, The First Affiliated Hospital of Bengbu Medical College, Bengbu, Anhui 233000, China

## Abstract

The incidence of prostate cancer is gradually increasing. There are many methods for clinical treatment of prostate cancer, such as surgical treatment and endocrine treatment. In the case of advanced prostate cancer, we must not only extend patients' survival times but also enhance their quality of life. Endocrine medications are the most effective therapy for advanced prostate cancer. This research will investigate the therapeutic impact of a complete treatment model in prostate cancer in order to discover a trustworthy clinical treatment model. This research discovered that, as compared to endocrine treatment, radical resection of prostate cancer may diminish and reach lower serum PSA levels in a short amount of time, as well as sustain low PSA levels and delay progression to castration resistance. Moreover, the comprehensive treatment mode can effectively reduce the possibility of complications. The research results show that the comprehensive treatment model can play an important role in the treatment of prostate cancer.

## 1. Introduction

Prostate cancer is the most common malignant tumor in Europe. China's prostate cancer ranks third in the male genitourinary system malignant tumor bureau. Internationally, endocrine therapy is still the main treatment for advanced prostate cancer. In China, we received adjuvant androgen deprivation treatment and orchiectomy. The results show that the combined application can reduce the incidence of tumor progression and improve the tumor-specific survival rate. This is true not just in cases of seminal vesicle invasion but also in cases of lymph node metastasis [1].

Prostate cancer (PC) incidence varies significantly by geography and ethnicity. PC is the most common kind of cancer in Europe and the United States, with a fatality rate second only to lung cancer. The incidence of PC in China is lower than that of the two countries, but it has shown a significant growth trend in recent years [2].

Among the malignant tumors of all organs, the natural history of PC has many changes. The tumors of most patients can be latent for a long time or even remain undetected for life. Radical surgery for PC is the main treatment for localized early prostate cancer. However, because the early symptoms of prostate cancer are hidden, once diagnosed, most patients have local or distant metastases, and there are few cases suitable for radical surgery. Prostate cancer in advanced stages is characterised by growing dysuria, urine retention, and metastatic symptoms, all of which pose a major danger to patients' quality of life and survival [3]. The endocrine therapy of PC has been used for more than 60 years, and it is still the main method for the current treatment of PC. Although the survival period of most patients is delayed, in the end, most advanced PCs appear hormone-independent or hormone-refractory. Other treatment methods include radiotherapy, chemotherapy, and immunotherapy. Although these treatments have certain curative effects, they also have obvious limitations. Therefore, the development of treatment methods for advanced PC, especially hormone-independent PC, has important clinical significance.

At present, regular prostate cancer screening has not been universal, and most elderly patients are already in the advanced stage when they are diagnosed and have lost the chance of cure. Most prostate cancer patients cannot be diagnosed because of the lack of obvious early symptoms, and the diagnosed prostate cancer patients often have advanced to the middle and advanced stages. The majority of them will develop hormone-independent type prostate cancer, also known as resistant prostate cancer, after surgery, conformal radiation and chemotherapy, and endocrine treatment. The most prevalent distant metastatic location for prostate cancer is the bone. Severe pain, pathological fractures, and signs of spinal nerve compression are the most common clinical findings. Pain not only has an impact on patients' quality of life but it also has an impact on their appetite, sleep, psychology, and therapeutic therapy. Currently, the western medicine treatment strategy for prostate cancer bone metastasis pain is mostly analgesics, but as the illness progresses and adverse responses to analgesics become more common, the effectiveness and usage of analgesics are substantially impacted. Traditional clinical practise has a lengthy history in long-term clinical practise. Chinese medicine workers have accumulated a lot of clinical experience in the treatment of cancer pain through internal use of traditional Chinese medicine, external treatment, acupoint application, and acupuncture, and achieved certain effects. At present, the treatment of bone metastasis pain of prostate cancer is often supplemented by traditional Chinese medicine to improve the symptoms of patients and improve their quality of life, which has shown gratifying therapeutic effects. There are many clinical studies on the efficacy and safety of integrated Chinese and Western medicine in the treatment of bone metastasis pain from prostate cancer, but there is a lack of large-sample, multicenter studies.

Prostate cancer is one of the most common malignant tumors that threaten the health of middle-aged and elderly men in the world. In the United States, the incidence of prostate cancer ranks first among male malignant tumors and ranks second among male cancer-related death rates. Compared with European and American countries, the incidence of prostate cancer in China is relatively low. However, with many factors such as changes in people's living habits, accelerating aging, and the gradual emphasis on prostate cancer screening, the incidence rate in China is showing a clear upward trend. In recent years, the rate of increase in the incidence of prostate cancer in China has even surpassed that of developed countries in Europe and America. In the United States, 80% of prostate cancer patients are diagnosed as early localized, and the proportion of locally advanced prostate cancer is only about 10%. As China's early prostate cancer screening system has not been perfected and popularized, the proportion of newly diagnosed patients with advanced prostate cancer in China is relatively high, and about one-third of newly diagnosed patients have progressed to locally advanced prostate cancer.

This paper explores the role of comprehensive treatment models in the treatment of prostate cancer, and provides a theoretical reference for the subsequent treatment effects of prostate cancer.

## 2. Related Work

With the improvement of surgical techniques and an in-depth understanding of the local anatomical characteristics of the prostate, radical prostatectomy has become a safe and effective treatment for prostate cancer [4]. This operation is suitable for patients with tumors younger than 73 years old, with good general conditions, localized, and stage B tumors and can improve the survival rate of some patients. Patients with well-differentiated tumours below stage B had 3-year and 7-year survival rates of 98.3% and 98.3%, respectively. Patients with moderately differentiated tumours had survival rates of 90.4 percent and 85.9%, respectively. Patients with poorly differentiated malignancies had survival rates of 84.8 percent and 54.4 percent, respectively. Patients with poorly differentiated malignancies have a worse survival percentage as time goes on [5]. The prognosis for stage A tumours has been regarded favourable, and aggressive surgery has not been recommended. Because stage B patients have a long life expectancy and the tumour is totally contained inside the prostate, radical prostatectomy should be done immediately to guarantee that all tumour tissue is removed. The impact is not favourable for people with stage C and D [6]. Retropubic radical resection of prostate cancer and transperineal radical resection of prostate cancer are the two basic types of radical prostatectomy. The operation requires the removal of the entire prostate, seminal vesicles, and pelvic lymph nodes on both sides and an anastomosis of the bladder neck and posterior urethra. Most urologists now advocate the use of the former, which has the advantage of a wide surgical field and the ability to clean the affected pelvic lymph nodes. The advantage of the transperineal route is that the surgical trauma is small, and the route to the local tumor is simple, which is conducive to the anastomosis of the urethra and the bladder neck. The most disturbing side effects of radical prostatectomy in the past are postoperative urinary incontinence and impotence. The former can be avoided as long as the technique of the anastomosis of the urethral stump retaining the external sphincter and the bladder neck is mastered [7]. Most patients may maintain normal sexual function following surgery because to advancements in sexual neuroprotection technologies. With the advancement and maturation of laparoscopic technology in recent years, video laparoscopy-assisted radical resection of early prostate cancer has become one of the standard surgical techniques for early prostate cancer. The majority of surgical indications are limited to TIbeT stage 2 patients inside the prostate capsule. It also has the benefits of causing less trauma, allowing patients to recover faster, and allowing for simultaneous pelvic lymph node dissection if required [8]. Many hospitals have started to perform laparoscopic radical prostatectomy using the Da Vinci robotic surgical equipment. The system is a well-established computer-assisted remote operating system. The surgical field of view is enlarged, operator's tiredness is decreased, involuntary jitter during manual operations is avoided, man-made pollution is minimised, and operation's precision and safety are increased [9]. Literature [10] reported that the robot-assisted laparoscopic radical prostatectomy group is equivalent to or better than the traditional surgery group. It has fewer postoperative complications, reduced intraoperative blood loss, and speeds up the process of beginners to master laparoscopic radical prostatectomy.

Due to the hidden incidence of prostate cancer, it is difficult to diagnose early, and advanced prostate cancer accounts for the majority. 90.2% of patients with advanced prostate cancer (C, D) have bladder outlet obstruction, and 41.5% have urinary retention [11]. In the past, suprapubic cystostomy was used to relieve the symptoms of urethral obstruction. The literature [12] used TURP to treat spreading prostate cancer, especially stage c lesions, and achieved good results. The literature [13] used TURP to treat urethral obstruction caused by advanced prostate cancer, and the effect is better. The literature [14] performed TURP therapy and endocrine therapy on prostate cancer patients with IPSS ≥ 15 points. Compared with endocrine therapy alone, the quality of life of the former group was significantly higher than that of the latter group. The results also support the above view. The literature [15] uses electrovaporization (TUVP) to treat prostate cancer. Compared with TURP, it has less bleeding, shorter operation time, and clear vision. The principle of plasma technology is that the working electrode and the return electrode of the bipolar electrosurgical are located in the electrosurgical ring, and the current does not need to pass through patient's body. The high-frequency electric energy forms a simplified local control circuit through the conductive saline solution, and a high-energy ion sphere is formed between the electrocutting working electrode and the attached circuit electrode. This plasma sphere has enough energy to break the organic molecular bonds (such as chemical bonds, hydrogen bonds, and ionic bonds) in the target tissue, so that the target tissue is cracked, broken, and vaporized [16]. Its characteristic is that the surface temperature of the target tissue is only 40-70°C, the cutting is accurate, and the heat penetration is shallow. Its unique feature is that it must produce an effect in the conductive liquid through a bipolar method and use physiological saline as the conductive liquid, so it is also called “plasma” technology. The characteristics of plasma technology are low surface tissue temperature, slight damage to surrounding tissues, and shallow heat penetration. Moreover, the radio frequency ion beam generator controller is intelligent, and the contact with the envelope during the electrode cutting process can stop the radio frequency energy transmission, generate a warning, and automatically protect the prostate envelope tissue. In addition, it has the characteristics of less bleeding. There are not many reports about plasma beam treatment of prostate cancer, but because plasma technology is safe and reliable, it may become a new way to replace traditional electrosurgical surgery [17]. Patients with stage C and D prostate cancer who are no longer candidates for radical resection and are above the age of 70 may benefit from endoprostatic treatment. These individuals have an anticipated life span of fewer than 10 years, and they have apparent symptoms such as lower urinary tract blockage or recurrent urinary tract infection, bleeding, urine retention, and obstructive renal insufficiency. The procedure not only eliminated the majority of the prostate disease tissue, but it also eased the posterior urethral blockage, and patient's subjective symptoms and quality of life improved dramatically. However, intracavitary treatment is only a palliative treatment measure, which can only relieve the symptoms of lower urinary tract obstruction but cannot cure prostate cancer. The treatment of advanced patients should be comprehensive treatment [18].

## 3. Materials and Methods

All patients selected in this paper underwent prostate biopsy, serum PSA test, digital rectal examination, prostate MRI examination, chest CT, abdominal ultrasound, and whole body bone imaging. During the treatment, the patients are followed up every month to understand their PSA changes, disease progression and adverse reactions during the treatment process.

The patients are determined comprehensively based on digital rectal examination, prostate MRI, transrectal prostate ultrasound, chest, abdomen and pelvic CT, puncture, pathology, and needle number distribution. The standard is based on AJCC 2010 version of prostate cancer TNM staging.

All patients have a transrectal ultrasonography prostate puncture and are given bowel preparation before measuring the diameters of the prostate glands up and down, front and back, left and right, and calculating the estimated volume of the glands using the formula: PV(ml) = 0.52∗diameters up and down∗diameters left and right∗diameters front and back cm A 12-needle puncture is standard, with an additional 1-2 needles inserted for patients who have nodules on ultrasonography. Antibiotics are given intravenously on a regular basis to avoid infection following the procedure. Two pathologists examine the abnormal sections and determine the main and subregional grades in order to calculate Gleason scores.

The three observation groups are as follows. The control group 1 receives continuous endocrine therapy. The control group 2 receives laparoscopic radical resection combined with endocrine therapy. The experimental group receives neoadjuvant endocrine therapy combined with laparoscopic radical resection [19].

Before venous blood collection, the patient has no ejaculation for 24 hours, no catheterization or cystoscopy for 48 hours, no digital rectal examination within 1 week, no prostate puncture within 1 month, and no history of acute prostatitis and urinary retention [20].

In order to understand the clinical effect of multimodal comprehensive therapy on patients with locally advanced prostate cancer, the clinical data during the treatment process and the perioperative period were used as observation indicators. The general clinical data of the first diagnosis include age, body mass index, serum PSA value, prostate volume, clinical stage, and puncture pathology. The curative effect observation indicators are the changes of serum PSA, urination, and quality of life scores and the proportion and time of progression to CRPC at 1, 6, and 12 months after treatment. Perioperative data includes operation time, intraoperative bleeding, postoperative hospital stay, catheter and drainage catheter removal time, surgical biochemical recurrence ratio, and complications data: rectal injury, lymphatic leakage, anastomotic leakage, and urinary incontinence. Postoperative pathology includes positive rate of resection margin, positive rate of regional lymph nodes, and postoperative Gleason score.

All of the patients in the cohort had laparoscopic radical prostatectomy, which senior specialists perform. The following are the major stages in the procedure. The patient is put in a supine posture once the general anaesthetic has worn off, and a 3 cm incision is made through the umbilicus in the centre of the lower abdomen to separate the posterior rectus abdominis sheath layer by layer. The extraperitoneal fat is bluntly separated with a finger, and a self-made balloon is used to inflate about 800 ml. After separating the gap, the patient inserts a 10 mm Trocar through the incision. The pressure of the pneumoperitoneum was set to 15 mmHg, and a 12 mm Trocar was placed on the left and right sides of the two transverse fingers under the umbilicus on the outer edge of the rectus abdominis under direct observation of the laparoscopic screen. If necessary, the patient needs to place a 5 mm Trocar at McDonald's point and the anti-McDonald's point and take the 150-300 head-high-foot-low position after the card is placed. After that, it is necessary to separate the pelvic floor fascia and the surface fat of the prostate, open the pelvic fascia and pubic prostatic ligament on both sides, and tie the dorsal deep venous complex with a figure of 8 with 3/0 barb line. After that, pelvic lymph node dissection is performed, and bilateral external iliac blood vessels and obturator lymph nodes are routinely dissected. Then, you need to fully expose the bladder neck, identify the bladder neck opening, open the front lip of the bladder neck, pull out the urinary catheter, and open the back lip of the bladder with blunt and sharp separation to reveal the seminal vesicles and vas deferens on both sides. At the same time, it is necessary to cut and lift the vas deferens to open the Free the Denonvilliers gap between the prostate and the rectum. The lateral ligaments on both sides are ligated and cut off with Hemolok to expose the urethra and cut off the deep dorsal vein complex and urethra on the side of the prostate, and the two sides of the prostate are separated to the apex along this gap. The bladder neck and urethra are sutured constantly using 2/O Weiqiao suture under the direction of the urine catheter (3, 5, 7, 9, 11, 1 point). The sutures are tightened and knotted, the airbag is filled with water and secured, and no active bleeding is examined after the 20 Fr three-chamber urine catheter is indwelled with urinary catheters. Normal saline is administered along the catheter to see whether there is any leakage, and seams are added if required. The specimens are put in the specimen bag and removed from the subumbilical incision, with the left and right pelvic drainage tubes in situ. The lesion is covered with hemostatic gauze, the pneumoperitoneum is sutured layer by layer using the microscope, and a pathological investigation is sent [21].

## 4. Result

The results of comparison of observational data of patients' efficacy are shown in Table 1.

One month after treatment, the average PSA value of surgical patients in the control group 2 is lower than that in the control group 1 and the test group, and there is a statistical difference. There is no significant difference in the average PSA value between the three groups in the third month after treatment. At 6 months and 12 months after treatment, the average PSA value of the control group 1 and the control group 2 is significantly higher than that of the test group. After 12 months of treatment, the average PSA value of the test group is significantly lower than that of the control group 1 and control group 2, and it is statistically significant (*P* < 0.05). During the follow-up, the patients in the test group reached the average lowest PSA value lower than those in the A and B groups, and there was a statistical difference (*P* = 0.009). During the follow-up, the proportion of patients who progressed to castration-resistant prostate cancer is not statistically different among the three groups. However, the time for patients to progress to the castration resistance stage is significantly shorter in the control group 1 than in the other two groups. On this basis, the following comparison only compares the data of the control group 2 and the test group.

The comparison of perioperative indicators and complications between the two surgical groups is shown in Tables 2–6.

The operation time of the experimental group is shorter than that of the control group 2, and the amount of blood loss and the number of blood transfusions are significantly lower than that of the control group. The differences between the two groups are statistically significant. However, there is no significant difference between the postoperative drainage tube placement time, indwelling catheterization time, and postoperative hospital stay between the two groups. There is no statistical difference in the proportion of urinary incontinence between the two groups of patients at 3 and 6 months after surgery.

## 5. Analysis and Discussion

Clinically, there are doubts about whether surgical treatment of locally advanced prostate cancer can completely remove the lesion and whether it will increase related complications. In the past, due to the high rate of positive surgical margins and the high incidence of postoperative complications, the guidelines did not recommend surgical treatment as the first choice for locally advanced prostate cancer. Locally advanced prostate cancer invades tissues and organs beyond the prostate capsule, resulting in severe local adhesions, disordered tissue architecture, and a limited operating area, increasing the complexity of the procedure and the risk of perioperative complications. The frequency of serious perioperative problems has steadily decreased as detection and treatment technology has increased, as has surgical expertise, and the local surgical resection of the main tumour of locally advanced prostate cancer has been repositioned. The European Urology Guidelines for the Diagnosis and Treatment of Prostate Cancer Recommendations for radical surgery for patients with locally advanced prostate cancer have been raised from the level 3 evidence level C recommendation to a strong recommendation. China's urology guidelines also recommend surgery for stage T3b-4 prostate cancer, but it requires multidisciplinary discussion, fully weighing patient's surgical risks and postoperative benefits, and rigorous screening before proceeding. If the tumor is not fixed to the pelvic wall or does not invade the urethral sphincter, a relatively small tumor can be treated with radical surgery combined with adjuvant treatment. In the study, it is found that in this study, patients in the surgical group are strictly selected according to the guidelines. There are more patients in the surgical treatment group with earlier clinical stages than in the endocrine therapy group, and the patients are younger and have a longer life expectancy. The advantages of radical mastectomy for patients with locally advanced prostate cancer are radical mastectomy can remove local lesions to maintain the PSA level at a low level, thereby having the greatest inhibitory effect on tumor micrometastasis, delaying tumor progression, reducing postoperative biochemical recurrence rate, and improving tumor-specific survival of patients. Moreover, radical mastectomy for locally advanced prostate cancer can well control the development of local tumors. Three months after the operation, patient's serum PSA is close to zero. Postoperative high level of PSA suggests that there may be residual tumors, a faster increase in PSA level indicates the possibility of distant metastasis, and a slow increase in PSA level may indicate local recurrence. This research discovered that, compared to endocrine treatment, radical resection of prostate cancer may diminish and reach lower serum PSA levels in a short amount of time and sustain low PSA levels and delay progression to castration resistance. The benefit of radical resection is that it aids in the appropriate staging and grading of tumour malignancy and guides follow-up treatment based on postoperative pathology. If no radical surgery is performed, clinical staging is the only way to assess the disease before initial treatment, but it mainly relies on digital rectal examination and imaging examination, which is difficult to accurately determine the extent of tumor malignancy and the extent of invasion. In the preoperative clinical staging of cases judged to be locally advanced prostate cancer, many postoperative pathological results are actually localized prostate cancer. This part of the patients can achieve the effect of complete tumor resection, and the prognosis is good.

In this study, patients in the neoadjuvant therapy group received endocrine therapy for 3-6 months before surgery, and a small number of patients had complete adhesion of the tumor to the rectum without gap boundaries. After 6-9 months of endocrine therapy, the size of patient's prostate shrinks, and the space between the anterior rectum and the prostate reappears, making it possible to completely remove the tumor. In addition, compared with the direct operation group, the operation time is significantly shorter and the intraoperative bleeding is less. In our study, the positive rates of postoperative pathological margins are higher in the two surgical groups, which may be related to the small sample size in this study. After neoadjuvant endocrine therapy, patients who do not undergo direct surgery at the anatomical level are clear about the anatomical level, which increases the difficulty of the operation, and the intraoperative adhesions are more obvious, which makes the tip and base resection incomplete and increases the possibility of positive margins. However, whether this adhesion and level of ambiguity is caused by adhesion to surrounding tissues at a later stage or caused by neoadjuvant endocrine therapy is still difficult to clearly define.

For patients with locally advanced prostate cancer, surgical operation may still remove the tumor. Surgery may assist the enhancement of the efficacy of complete therapy by reducing tumour burden and increasing local control. When comparing the treatment effects of surgery-based comprehensive treatment and radical radiotherapy for patients with locally advanced prostate cancer, it was discovered that patients in the surgery group had significantly longer biochemical progression-free survival and overall survival than those in the radiotherapy group. Our investigation, on the other hand, found no significant differences. There is also research that neoadjuvant endocrine can improve the progression-free survival and overall survival of patients with locally advanced prostate cancer. However, most clinical studies currently lack long-term randomized controlled studies with endocrine therapy alone. For patients with locally advanced prostate cancer, the long-term efficacy of neoadjuvant therapy combined with radical prostatectomy remains to be seen. In this study, the survival analysis of the three groups of patients after continued follow-up is yet to be performed to observe the impact of different treatment methods on the long-term prognosis of patients.

## Figures and Tables

**Table 1:** Comparison of observation data of patients' curative effect.

	Control group 1	Control group 2	Test group
PSA after 1 month (ng/ml)	16.42 ± 32.17	1.64 ± 2.758	1.057 ± 8.33
PSA after 3 months (ng/ml)	4.76 ± 13.53	1.23 ± 1.53	2.15 ± 1.17
PSA after 6 months (ng/ml)	3.02 ± 3.89	0.55 ± 0.95	0.09 ± 0.56
PSA after 12 months (ng/ml)	1.95 ± 3.17	0.21 ± 0.32	0.03 ± 0.02

**Table 2:** Statistical table of operation time (min).

No.	Control group 2	Test group	No.	Control group 2	Test group
1	219.91	133.23	14	159.71	139.83
2	318.04	143.42	15	272.11	139.71
3	154.68	162.42	16	203.58	200.88
4	188.02	150.36	17	150.91	229.60
5	221.12	223.02	18	326.67	184.81
6	302.48	236.44	19	298.56	229.49
7	262.89	200.63	20	285.36	150.79
8	220.95	174.69	21	241.11	223.79
9	213.89	229.28	22	304.76	253.74
10	160.48	259.93	23	213.06	223.44
11	154.27	132.49	24	231.11	115.65
12	206.67	155.55	25	282.79	252.17
13	261.73	159.23			

**Table 3:** Statistical table of blood loss (ml).

No.	Control group 2	Test group	No.	Control group 2	Test group
1	361.66	244.47	14	333.33	321.63
2	382.13	181.85	15	284.19	413.59
3	251.59	267.76	16	320.02	440.80
4	439.63	372.00	17	460.97	135.25
5	269.30	446.40	18	491.46	406.41
6	533.81	439.48	19	262.88	233.94
7	298.70	107.07	20	526.02	443.24
8	379.80	429.97	21	283.73	92.29
9	518.04	203.99	22	303.20	279.14
10	386.15	93.18	23	312.70	377.95
11	258.14	101.86	24	418.64	420.20
12	269.26	393.78	25	408.43	200.67
13	317.83	417.31			

**Table 4:** Statistical table of drainage tube time (day).

No.	Control group 2	Test group	No.	Control group 2	Test group
1	7.70	13.46	14	11.54	13.26
2	8.93	9.75	15	7.08	12.54
3	11.53	9.34	16	4.76	10.91
4	5.39	11.84	17	6.28	7.82
5	11.93	9.93	18	4.99	9.40
6	7.41	13.65	19	11.86	9.44
7	8.43	13.33	20	11.42	6.45
8	8.12	7.21	21	6.72	9.46
9	8.35	6.59	22	10.26	6.73
10	11.32	11.37	23	7.46	7.76
11	7.31	5.98	24	12.27	13.11
12	5.29	10.83	25	11.78	10.50
13	11.84	8.68			

**Table 5:** Statistical table of catheterization time (day).

No.	Control group 2	Test group	No.	Control group 2	Test group
1	25.31	24.45	14	19.58	12.60
2	16.63	14.73	15	21.76	15.17
3	13.36	24.10	16	25.25	21.61
4	22.71	13.58	17	25.12	21.26
5	22.72	20.92	18	13.95	18.79
6	23.50	20.96	19	18.29	16.13
7	14.56	17.83	20	24.50	14.61
8	19.64	23.13	21	19.44	19.04
9	16.19	21.01	22	18.29	18.25
10	14.25	19.86	23	18.10	17.78
11	11.95	20.96	24	19.46	15.72
12	21.62	18.68	25	17.16	14.84
13	11.78	16.95			

**Table 6:** Statistical table of the number of days of hospitalization after operation (day).

No.	Control group 2	Test group	No.	Control group 2	Test group
1	11.96	7.33	14	5.88	5.56
2	7.23	8.56	15	19.68	9.86
3	20.50	10.92	16	21.40	7.92
4	6.25	6.60	17	12.91	7.79
5	10.05	5.83	18	17.46	11.04
6	10.18	11.79	19	18.85	14.14
7	11.60	6.08	20	12.44	13.92
8	12.57	10.74	21	10.87	10.64
9	9.19	7.05	22	9.98	8.34
10	14.61	12.81	23	17.54	6.87
11	6.04	9.69	24	6.37	11.61
12	15.72	11.79	25	12.84	9.24
13	18.78	11.84			

## Data Availability

The data used to support the findings of this study are included within the article.
